# Vitamin C and asthma in children: modification of the effect by age, exposure to dampness and the severity of asthma

**DOI:** 10.1186/2045-7022-1-9

**Published:** 2011-08-25

**Authors:** Harri Hemilä, Mohammed Al-Biltagi, Ahmed A Baset

**Affiliations:** 1 Department of Public Health, University of Helsinki, Helsinki, Finland; 2 Department of Paediatrics, Faculty of Medicine, Tanta University, Tanta, Gharbia Governorate, Egypt

**Keywords:** age factors, ascorbic acid, asthma, child, effect modifiers, forced expiratory volume, obstructive lung diseases, quality of life, controlled trials

## Abstract

**Background:**

We previously found a significant benefit of vitamin C supplementation in asthmatic children.

**Purpose:**

To test whether the effect of vitamin C on asthma is heterogeneous over the participant population.

**Methods:**

Egyptian asthmatic children between 7 and 10 years of age (n = 60) were included in the cross-over trial. They were administered 0.2 grams per day of vitamin C and placebo for separate 6-week periods. The variation in the vitamin C effect on two clinically relevant outcomes was analyzed: the childhood asthma control test (C-ACT), which measures the severity of asthma symptoms (the scale ranges from 0 to 27 points, < 20 points indicating unsatisfactory asthma control), and FEV_1_. We used linear modeling to examine the variation of the vitamin C effect in the subgroups.

**Results:**

The effect of vitamin C on the C-ACT was significantly modified by age and baseline C-ACT levels. In the children aged 7.0-8.2 years with a baseline C-ACT of 18 to 19 points, vitamin C increased the C-ACT score by 4.2 points (95% CI: 3.3-5.3); whereas in the children aged 8.3-10 years who had a baseline C-ACT of 14 to 15 points, vitamin C increased the C-ACT score by only 1.3 points (95% CI: 0.1-2.5). The effect of vitamin C on the FEV_1 _levels was significantly modified by age and exposure to dampness. In the children aged 7.0-8.2 years with no exposure to dampness, vitamin C increased the FEV_1 _level by 37% (95% CI: 34-40%), whereas in the children aged 8.3-10 years with exposure to dampness or mold in their bedroom more than one year prior to the study, vitamin C increased the FEV_1 _level by only 21% (95% CI: 18-25%).

**Conclusions:**

We found strong evidence that the effect of vitamin C on asthmatic children is heterogeneous. Further research is needed to confirm our findings and identify the groups of children who would receive the greatest benefit from vitamin C supplementation.

## Background

Proposals that vitamin C might be beneficial in the treatment of asthma date back to the 1940s [1,2]. Nevertheless, the role of vitamin C is still undefined. A study of Nigerian asthmatics reported a 78% lower incidence of asthma attacks in those administered vitamin C [3], whereas a study of British asthmatics found no effect of vitamin C on the symptoms or on the FEV_1 _levels [4]. Three trials found that vitamin C reduces bronchoconstriction caused by exercise in subjects who suffer from exercise-induced bronchoconstriction (EIB) [5-7]. Although these three EIB studies imply that vitamin C may have an effect on lung function, the findings cannot be generalized to patients with other variants of asthma.

There is no well-defined mechanism whereby vitamin C may have an effect on asthma. Nevertheless, vitamin C influences the production of various prostanoids in lung tissues [8-11]. Indomethacin reverses the effect of vitamin C on bronchoconstriction in guinea pigs [10-13] and humans [14,15]. Thus, the effect of vitamin C on airways might be, at least partly, mediated by influences on the prostanoid metabolism. Furthermore, in asthmatic patients, the level of vitamin C is low in plasma [1,16-18] and bronchoalveolar fluid [19]. Although such a correlation does not imply a causal relationship, it encourages research on vitamin C and asthma.

We have previously carried out a placebo-controlled cross-over trial in which we examined the effect of vitamin C, zinc, omega-3 fatty acids and their combination in Egyptian asthmatic children [20]. Vitamin C significantly decreased asthma symptoms and increased the FEV_1 _levels [20]. We reasoned that the effect of vitamin C might be greater in children who had low baseline FEV_1 _levels and found that the effect was modified by baseline FEV_1 _(unpublished). Therefore we decided to carry out a formally planned subgroup analysis of the data.

In this subgroup analysis, we planned to use two clinically relevant outcomes: asthma symptoms as measured by the childhood asthma control test (C-ACT) [21,22] and pulmonary function as measured by FEV_1_. We planned to examine the effect of six baseline variables: the C-ACT, the FEV_1_/FVC ratio, gender, paternal smoking, exposure to dampness or mold in the bedroom, and residential neighborhood. In this subgroup analysis, we decided to use the baseline FEV_1_/FVC ratio instead of the baseline FEV_1 _since the former adjusts for the variation in the size of lungs.

## Methods

### Participants and study design

The design and methods of the trial have been described earlier [20]. In brief, 72 Egyptian children between 7 and 10 years of age, who were diagnosed of having moderate persistent asthma (see [21] for the diagnostic criteria), were included in the trial. Twelve children were lost at follow-up due to change in their residence. This study reports the findings of the remaining 60 children (Table 1). The study was a randomized, double-blind, placebo-controlled cross-over trial carried out over 38 weeks. After a pre-trial assessment period of 2 weeks, the children entered the study on their normal diet, after which they entered five different 6-week therapeutic phases in a random sequence, with observers, participants and families blinded to the treatment: placebo, vitamin C, zinc, omega-3 fatty acids, and a combination of the three. Each phase was followed by a 2-week washout period before the next phase. Thus, by the end of the study, all the children had been exposed to the five treatment phases (placebo included) but in different sequences. In the vitamin C phase, the children were administered 0.2 g per day of ascorbic acid in capsules that appeared identical to the placebo capsules. The trial was approved by the Department Council and the Faculty Ethical committee. The current subgroup analysis is restricted to the comparison of the vitamin C and placebo phases.

**Table 1:** Demographic data of the asthma patients

Number of children who started the trial	76
Number of children who completed the trial	60

	Mean (SD)

Age (yr)	8.4 (1.0)

Weight (kg)	32 (18)

Height (cm)	124 (21)

BMI (kg/m^2^)	17.2 (1.3)

	No. of children

Boys/Girls	38/22

Urban/Rural	34/26

Associated nasal allergy	12

Asthma medications:	

Long acting β_2_-agonist alone	0

Moderate daily dose inhaled corticosteroid	16

Long acting β_2_-agonist + inhaled corticosteroid	20

β_2_-agonist + inhaled corticosteroid + intermittent short acting β_2_-agonist	18

β_2_-agonist + inhaled corticosteroid + sodium cromoglycate	6

Allergy medications:	

Antihistamine	24

Intermittent nasal decongestant	24

Nasal corticosteroid	16

### Background data and outcomes

At the beginning of the study and at the end of each treatment phase, the severity of asthma was assessed using the childhood asthma control test (C-ACT), and a pulmonary function test was performed. The C-ACT is a questionnaire for asthmatic children and their parents for identifying children aged 4-11 years whose asthma is inadequately controlled: the scale ranges from 0 to 27 points, < 20 points indicating unsatisfactory asthma control [22,23]. Spirometry was performed in a sitting position by all the children (spirometer: Morgan TLC Test Mk 11, Morgan Scientific, Haverhill, MA, USA). Participants performed three acceptable FVC maneuvers, and the highest FEV_1 _value was recorded.

Information on the presence of dampness or mold in the bedroom was obtained with a questionnaire based on four items confirmed by parent reporting [24]: 1) mold odor (n = 3), 2) visible mold (n = 29), 3) moisture (n = 19), 4) water damage (n = 21). Dampness or mold in the bedroom was defined as one or more positive responses. The question about the time of exposure to dampness had two alternatives: 1) "during the past 12 months" and 2) "only earlier" (*i.e*. more than one year prior to the study); only one child chose both the recent and earlier exposure alternatives.

As the outcome for the FEV_1 _change, we calculated the percentage increment in the FEV_1 _value between the end of the vitamin C and placebo phases. As the primary outcome for the C-ACT change, we calculated the arithmetic difference in the C-ACT between the end of the vitamin C and the placebo phases. Since we found that the vitamin C effect on the C-ACT was greater on participants with high baseline C-ACT values (Table 2), in Table 3 we also calculated the percentage increment in the C-ACT scores as a secondary outcome. In the normal plot, the distribution of the changes in the C-ACT and FEV_1 _were quite close to the normal distribution.

**Table 2:** Effect of vitamin C on the symptoms of asthmatic children

Subgroup	No. of Children	C-ACT (mean)		Difference in C-ACT		Test for interaction (P)
			
		Placebo	Vitamin C	Estimate	95% CI	
All	60	16.57	19.60	3.03	2.53-3.54	

C-ACT at baseline						

13-15	30	15.8	18.1	2.3	1.7-3.0	0.004^a)^
	
16-19	30	17.3	21.1	3.7	3.0-4.5	

FEV_1_/FVC (%)						

< 59	28	16.4	19.3	2.9	2.3-3.6	0.7^a)^
	
≥59	32	16.8	19.9	3.1	2.3-3.9	

FEV_1 _at baseline (L/s)						

< 1.1	29	16.7	20.3	3.6	3.0-4.3	0.013^a)^
	
≥1.1	31	16.5	18.9	2.5	1.7-3.2	

Age (yr)						

7.0-8.2	30	16.6	20.3	3.7	3.1-4.3	0.004^a)^
	
8.3-10	30	16.5	18.9	2.3	1.5-3.1	

Weight (kg)						

23-28	29	16.6	19.3	2.7	1.9-3.5	0.2^a)^
	
29-37	31	16.6	19.9	3.3	2.7-4.0	

Gender						

Girl	22	16.5	19.5	3.0	2.2-3.9	1.0
	
Boy	38	16.6	19.6	3.0	2.3-3.7	

Dampness exposure						

Never	25	16.8	19.2	2.4	1.4-3.4	0.1^b)^
	
During past 1 yr	20	16.3	19.7	3.4	2.6-4.2	

Earlier	14	16.5	20.1	3.6	2.8-4.4	

Smoking by the father						

Never	21	16.5	19.0	2.5	1.6-3.5	0.4^c)^
	
Current	22	16.8	19.8	3.0	2.2-3.9	

Ex-smoker	17	16.4	20.0	3.6	2.7-4.6	

Residential area						

Urban	34	16.5	19.5	3.0	2.4-3.7	1.0
	
Rural	26	16.7	19.7	3.0	2.2-3.9	

a) The test of interaction was calculated by using dichotomized variables for the C-ACT, FEV_1_/FVC ratio, FEV_1_, age, and weight (cut points at the medians). The test of interaction by using the continuous variables gives P = 0.0002 for the baseline C-ACT and P = 0.005 for age.

b) The test of interaction is restricted to the "Never" and "During past 1 yr" subgroups. One child who was exposed to dampness both "During past 1 yr" and "Earlier" is excluded from this subgroup comparison.

c) The test of interaction is restricted to the "Never" and "Current" subgroups.

**Table 3:** Vitamin C and asthma symptoms: effect modification by age and baseline asthma severity

Age (yr)	C-ACT at baseline	No of. Children	Symptoms (C-ACT) Mean		Arithmetic increase in C-ACT^a)^		Percentage increment in C-ACT^b)^	
			
			Placebo	Vitamin C	Mean	95% CI	Mean	95% CI
7.0-8.2	18-19	12	17.6	21.8	4.2	3.3-5.2	24%	18-31%
	
	16-17	10	16.3	20.0	3.7	2.4-5.0	23%	15-32%
	
	13-15	8	15.5	18.5	3.0	2.4-3.6	19%	16-23%

8.3-10	18-19	8	17.2	21.0	3.7	1.6-5.8	23%	9-36%
	
	16-17	10	16.8	19.2	2.4	1.5-3.3	14%	9-20%
	
	14-15	12	15.8	17.2	1.3	0.1-2.5	9%	1-17%

a) Arithmetic increase in the C-ACT. When age and baseline C-ACT as continuous variables were included in the linear model explaining the effect of vitamin C, the model was improved by χ^2^(2 df) = 19.1, P = 0.00007 (model parameters are shown in Table 4). There was no second order interaction between the baseline C-ACT and age in their modification of the vitamin C effect (χ^2^(1 df) = 2.1, P = 0.2).

b) Percentage increment in the C-ACT. When age and baseline C-ACT as continuous variables were included in the linear model explaining the effect of vitamin C, the model was improved by χ^2^(2 df) = 14.0, P = 0.0009. There was no second order interaction between the baseline C-ACT and age in their modification of the vitamin C effect (χ^2^(1 df) = 2.6, P = 0.1).

### Statistical methods

To minimize the multiple comparison problem associated with subgroup analysis, we wrote a protocol in which we planned this study (Additional file 1). We decided to focus on two clinically relevant primary outcomes, the C-ACT difference and the FEV_1 _ratio (above), and to examine the possible modification of the vitamin C effect by six variables: the baseline C-ACT, the baseline FEV_1_/FVC ratio, gender, paternal smoking, dampness or mold in the bedroom, and residential neighborhood (urban/rural) (see details in the Additional file 1). This series of subgroup analyses were motivated by our finding that the baseline FEV_1 _modified the vitamin C effect on the FEV_1 _level. In the subgroup analysis protocol, we considered that the baseline FEV_1_/FVC ratio would be a better variable for subgroup division as it adjusts for the size of the lungs. Unexpectedly, we did not find a modification of the vitamin C effect by the baseline FEV_1_/FVC ratio. The baseline FEV_1 _has a close correlation with age (r = 0.95), whereas the correlation between the baseline FEV_1 _and the baseline FEV_1_/FVC ratio is weak (r = 0.12). Therefore, we added FEV_1 _and age to the tables to examine whether the divergence between the baseline FEV_1_/FVC ratio and the FEV_1 _levels might be explained by age. Furthermore, we also added weight to the tables to test whether it is the young age *per se *or the low weight (higher dose per weight unit) that better explains the greater effect on the younger children.

We divided the children into subgroups by C-ACT, FEV_1_/FVC ratio, FEV_1_, age, and weight with the cut points at the medians. Effect modification by paternal smoking was tested by comparing never smokers with current smokers, so that ex-smokers were excluded. Similarly, effect modification by dampness or mold in the bedroom was tested by comparing never exposed to those children who were only recently exposed (< 1 year), so that those exposed to dampness in their earlier childhood (> 1 year prior to the study) were excluded. The excluded groups are shown in the tables, but they were not included in the test of interaction.

We tested the interaction between vitamin C effect and the subgroup variables by using linear models. To test whether the vitamin C supplementation effect is different between the subgroups, we first added a uniform vitamin C effect to all the children. Then we added an interaction term between vitamin C and the subgroup variable. The improvement of the linear model fit was thereafter calculated from the change in -2 × log (likelihood), which follows the χ^2 ^distribution with degrees of freedom defined by the number of interaction terms.

Although the C-ACT difference was close to the normal distribution, the values were integers in a range of -2 to +6 points. Therefore, we confirmed the most essential subgroup differences in Table 2 by a nonparametric test. The Wilcoxon test gave similar P-values for the interaction test between vitamin C effect on C-ACT and the dichotomous baseline C-ACT (P = 0.010) and age (P = 0.005), consistent with the t-test results in Table 2. The linear models, the t-test-based 95% confidence intervals (95% CI) of the effects, and the Wilcoxon tests were calculated using the R-package [25]. Two-tailed P-values are shown.

## Results

The essential characteristics of the 60 children are described in Table 1. On average, vitamin C supplementation increased the asthma symptom score, C-ACT, by 3.0 points (Table 2). This effect was modified by the baseline C-ACT so that vitamin C was more effective in those children who had less severe asthma symptoms. The evidence of effect modification was stronger when the baseline C-ACT was included in the statistical model as a continuous variable (P = 0.0002) than as a dichotomous variable (P = 0.004), which indicates that the effect modification was better captured by the continuous baseline C-ACT.

The baseline FEV_1_/FVC ratio did not modify the effect of vitamin C on the C-ACT (Table 2). This was inconsistent with the modification caused by the baseline FEV_1_, which gave us the motivation for this subgroup analysis. Because of this discrepancy, we considered that the modification by the baseline FEV_1 _might be explained by the close correlation between age and FEV_1_. Since age significantly modified the vitamin C effect, whereas baseline FEV_1_/FVC ratio did not, we concluded that the modification by the baseline FEV_1 _was simply reflecting the effect of age on FEV_1 _(Table 2). There was no substantial difference between including age as a dichotomous or a continuous variable in the statistical model. Gender and residential area did not modify the effect of vitamin C. There was also no significant difference between the children who were currently or had never been exposed to dampness in the bedroom, or between the children whose fathers were current smokers or had never smoked (Table 2).

Given that the baseline C-ACT and age modified the effect of vitamin C, we analyzed the combined effect of these two variables (Tables 3 and 4). When both of these variables were simultaneously included in the linear model, it was substantially improved (P = 0.0001), so that the proportion of variance in the vitamin C effect explained by these two variables was 27% (R^2 ^= 0.27). There was no second order interaction between these two variables in their influence on the vitamin C effect (Table 3). The greatest effect of vitamin C on the C-ACT was seen in the younger children who had mild asthma symptoms (4.2 point increase), whereas the smallest effect was seen in the older children who had severe asthma symptoms (1.3 point increase). The estimated influence of the baseline C-ACT and age on the vitamin C effect is shown in Table 4.

**Table 4:** Effect of vitamin C on the C-ACT level: parameters estimating the effect modification by age and baseline C-ACT

Variable	Effect of vitamin C on the C-ACT level^a)^
Age 7.0 yr, baseline C-ACT 13 points	+2.12 (SE 0.65)

Age (per year over 7.0 yr)	-0.52 (SE 0.22)

Baseline C-ACT (per point over 13)	+0.46 (SE 0.13)

a) These parameters are from the linear model for the arithmetic increase in C-ACT described in the footnote of Table 3. SE, standard error. This model predicts, for example, that a 9-yr old child with baseline C-ACT of 19 would have 3.84 point increase in C-ACT by vitamin C administration which is close to that observed (3.7) for the older children with baseline C-ACT 18 or 19 in Table 3.

In our analysis of the C-ACT change, we used the absolute difference as the primary outcome. However, as we found a greater effect in those children who had a high initial C-ACT score, we also analyzed Table 3 heterogeneity by using the percentage increment in the C-ACT score. With this secondary outcome, we also found strong evidence of heterogeneity in vitamin C effect between the children (P = 0.001).

On average, vitamin C increased the FEV_1 _level by 29% (Table 5). This effect was modified by age, and continuous age was better than dichotomous age in capturing the interaction (Table 5). The effect of vitamin C on FEV_1 _was also modified by dampness in the bedroom. Our test of interaction was restricted to the children who were currently or had never been exposed to dampness in the bedroom. However, the effect of vitamin C was smallest in the children who were exposed to dampness in their earlier childhood. Other tested baseline variables did not modify the effect of vitamin C (Table 5).

**Table 5:** Effect of vitamin C on the FEV_1 _levels of asthmatic children

Subgroup	No. of Children	FEV_1_ Mean (L/s)		Change in FEV_1_		Test for interaction (P)
			
		Placebo	Vitamin C	Estimate	95% CI	
All	60	1.125	1.446	28.9%	27.3-30.4%	

C-ACT at baseline						

13-15	30	1.16	1.48	27.5%	25.4-29.6%	0.07^a)^
	
16-19	30	1.09	1.41	30.3%	28.0-32.6%	

FEV_1_/FVC (%)						

< 59	28	1.11	1.43	29.4%	27.0-31.9%	0.5^a)^
	
≥59	32	1.14	1.46	28.4%	26.3-30.5%	

FEV_1 _at baseline (L/s)						

< 1.1	29	1.00	1.31	31.1%	28.6-33.6%	0.004^a)^
	
≥1.1	31	1.24	1.58	26.8%	25.1-28.5%	

Age (yr)						

7.0-8.2	30	1.00	1.31	31.1%	28.7-33.5%	0.003^a)^
	
8.3-10	30	1.25	1.58	26.7%	24.9-28.4%	

Weight (kg)						

23-28	29	1.12	1.44	29.7%	27.1-32.3%	0.3^a)^
	
29-37	31	1.13	1.45	28.1%	26.2-30.0%	

Gender						

Girl	22	1.07	1.37	28.6%	25.6-31.6%	0.8
	
Boy	38	1.16	1.49	29.0%	27.2-30.9%	

Dampness exposure						

Never	25	1.16	1.53	32.4%	30.2-34.6%	0.001^b)^
	
During past 1 yr	20	1.11	1.42	27.6%	25.9-29.4%	

Earlier	14	1.07	1.34	25.0%	21.2-28.8%	

Smoking by the father						

Never	21	1.17	1.52	30.1%	28.0-32.2%	0.4^c)^
	
Current	22	1.08	1.38	28.5%	25.3-31.7%	

Ex-smoker	17	1.12	1.43	27.9%	24.9-30.9%	

Residential area						

Urban	34	1.09	1.40	29.2%	27.2-31.3%	0.6
	
Rural	26	1.17	1.50	28.4%	25.8-31.0%	

a) The test of interaction was calculated by using dichotomized variables for the C-ACT, FEV_1_/FVC ratio, FEV_1_, age, and weight (cut points at the medians). The test of interaction by using the continuous variables gives P = 0.2 for the baseline C-ACT and P = 0.001 for age.

b) The test of interaction is restricted to the "Never" and "During past 1 yr" subgroups. One child who was exposed to dampness both "During past 1 yr" and "Earlier" is excluded from this subgroup comparison.

c) The test of interaction is restricted to the "Never" and "Current" subgroups.

When both age and exposure to dampness were included in the same statistical model to explain FEV_1 _changes, the model was significantly improved (P = 10^-10^) (Tables 6 and 7). The proportion of variance in the vitamin C effect explained by the two variables was 58% (R^2 ^= 0.58). There was no second order interaction between age and exposure to dampness in their influence on the vitamin C effect. The greatest effect of vitamin C on FEV_1 _was seen in the younger children who had never been exposed to dampness or mold in their bedroom (37% increase in FEV_1_), whereas the smallest effect was seen in the older children who had been exposed to dampness more than one year prior to the study (21% increase in FEV_1_)(Table 6). The estimated influence of age and exposure to dampness on the vitamin C effect is shown in Table 7.

**Table 6:** Vitamin C and FEV_1_: effect modification by age and exposure to dampness

Age (yr)	Exposure to dampness in the bedroom	No of. Children^a)^	FEV_1 _(L/s)		Percentage increment in FEV_1 _^b)^	
			
			Placebo	Vitamin C	Mean	95% CI
7.0-8.2	Never	10	0.98	1.34	37.0%	33.9-40.2%
	
	During past 1 yr	11	1.04	1.34	29.0%	27.4-30.6%
	
	Earlier	9	0.99	1.25	27.1%	21.5-32.6%

8.3-10	Never	15	1.28	1.66	29.3%	27.6-31.1%
	
	During past 1 yr	9	1.21	1.52	25.9%	22.5-29.4%
	
	Earlier	5	1.23	1.49	21.3%	18.0-24.5%

a) Since the goal of this table is to compare the effect of "During past 1 yr" and "Earlier" exposure to dampness, one child who had both modes of exposure was excluded (age 8.4 yr), making the number of children in this analysis 59.

b) When age as a continuous variable and the three categories of dampness were included in the linear model explaining the effect of vitamin C on the FEV_1 _increase, the model was improved by χ^2^(3 df) = 51.8, P = 10^-10 ^(model parameters are shown in Table 7). There was no second order interaction between age and dampness in their modification of the vitamin C effect (χ^2^(2 df) = 2.3, P = 0.3).

**Table 7:** Effect of vitamin C on the FEV_1 _level: parameters estimating the effect modification by age and exposure to dampness

Variable	Effect of vitamin C on the FEV_1 _level^a)^
Age 7.0 yr, no exposure to dampness	+37.9% (SE 1.2%)

Age (per year over 7.0 yr)	-3.37% (SE 0.52%)

Exposure to dampness during past 1 yr	-5.8% (SE 1.2%)

Exposure to dampness earlier	-9.6% (SE 1.4%)

a) These parameters are from the linear model described in the footnote of Table 6. SE, standard error. This model predicts, for example, that a 9-yr old child with exposure to dampness earlier than 1 year before the study would have 21.5% increase in FEV_1 _by vitamin C administration which is close to that observed (21.3%) for the older children with early dampness exposure in Table 6.

Since exposure to dampness was composed of four indicator items, we explored whether there might be differences between the indicators; mold odor was reported only by 3 children, and it was excluded from this comparison. Within the accuracy of the confidence intervals, there were no differences between the three other indicators in the modification of the vitamin C effect on the FEV_1 _level (data not shown).

## Discussion

We found that age modified the effect of vitamin C on asthma symptoms (C-ACT) and on the FEV_1 _level in this group of Egyptian children. In addition, the vitamin C effect on asthma symptoms was modified by baseline C-ACT, and the vitamin C effect on the FEV_1 _level was modified by exposure to dampness in the bedroom.

Previously, an age-dependent variation in the vitamin C effect on common cold duration was noted, but it was not evident whether the greater effect on children than on adults was caused by age *per se *or by a higher dose per weight unit since children weigh less [26,27]. In the current study, we found a greater vitamin C effect on younger children, and this was not explained by weight differences (Tables 2 and 5). Still, it is possible that the heterogeneity over age might be caused by some factors closely correlated with age; however, this possibility does not challenge the strong evidence indicating that substantial heterogeneity exists across this group of children.

When planning this subgroup analysis, we reasoned that the effect of vitamin C might be greater in children who had the lowest baseline C-ACT level and FEV_1_/FVC ratio, and in children who had been exposed to dampness (Additional file 1). However, we found the opposite direction for the modification by C-ACT, namely the effect of vitamin C was greater in those who had a high baseline C-ACT level. We also found that the relation between the baseline FEV_1 _and the vitamin C effect, which gave us the motivation for this study, was explained by age and not by the baseline FEV_1_/FVC ratio. In addition, contrary to our expectation, exposure to dampness in the bedroom was associated with a decreased effect of vitamin C. Thus, although the baseline C-ACT and dampness modified the vitamin C effect, the modification was in a direction opposite to our expectation.

Gender differences have been found in the vitamin C effects on the common cold [28-30], but in this study we did not find any differences between boys and girls. Urban and rural neighborhoods differ in the type of outdoor air pollution, and passive smoking causes irritation of the airways, but we found no modification of the vitamin C effect by residential neighborhood or paternal smoking.

We found substantial heterogeneity in the effect of vitamin C, over two-fold variation in the effect between the extremes of the subgroups in Tables 3 and 6. Thus, the effect of vitamin C on asthma seems to be context dependent. This heterogeneity in the vitamin C effect seems important since it indicates that no universal effect should be sought. Instead, the characteristics and living conditions of asthma patients who would get the greatest benefit from vitamin C should be targeted.

The heterogeneity we found within these children also has implications for the interpretation of previous studies. Two randomized, double-blind, placebo-controlled trials found divergent effects of vitamin C in asthmatic patients. In Nigeria, Anah et al. found a 78% reduction in the incidence of asthma attacks in 15 to 46 year-old patients administered 1 g/day of vitamin C [3]. In the UK, Fogarty et al. did not find any effect of 1 g/day of vitamin C on asthma symptoms or FEV_1 _levels in 18 to 64 year-old asthmatics [4]. Since differences in nutrition or lifestyle, or other differences between the participants of the two trials may explain the divergent findings, the newer trial [4] should not be considered a refutation of the older trial [3].

Asthma is a collection of different phenotypes, rather than a single disease [31,32]. These phenotypes are categorized under the broad umbrella of "asthma" because they meet the criteria for the clinical diagnosis of the disease. Allergic sensitization that triggers asthma may be the largest phenotype. There is also evidence that molds are an important environmental trigger for asthma exacerbations, and the effects of molds are possibly caused, at least partly, by their mycotoxins [24,33-35]. Furthermore, the mechanisms behind EIB seem to be different from those of ordinary asthma [36]. Given the variety of mechanisms causing asthma-type symptoms, it seems plausible that vitamin C has different effects on different types of asthma. Thus, although three trials consistently found a benefit of vitamin C against EIB [5-7], those studies cannot be extrapolated to other types of asthma. In this study, we found that the effect of vitamin C on the FEV_1 _level of asthmatic children was significantly modified by exposure to dampness or mold in the bedroom.

A number of subgroup comparisons were carried out in our study, and therefore the multiple comparison problem might be of concern. However, the particularly low P-values seen in Tables 2 and 5 are not easily explained by the 18 subgroup comparisons in these two tables. Furthermore, the proportion of variance in the vitamin C effect explained by the statistical models (R^2^) in Tables 3 and 6 is high. Therefore, we do not consider that the differences identified might be easily explained by multiple testing.

Our study was randomized, double blind and placebo controlled. Nevertheless, our study has various limitations. Our study subjects were Egyptian children, and it is not clear whether the same modifying factors might apply to children in industrialized countries or in other developing countries or to adults. There may have been inaccuracy in the measurement of mold exposure; however, nondifferential misclassification would move the estimate of interaction effect towards the null value (of no interaction) and cannot generate an artificial difference between the exposed and unexposed [37]. The duration of vitamin C administration was only 6 weeks, and it is not evident whether the observed effect lasts substantially longer. In a cross-over study, the carry-over effect from the intervention phase to the placebo phase could reduce the difference between the two phases, but cannot bias in the direction of greater effect. The dose of vitamin C was rather low, 0.2 g/day, and our study does not give any information about dose dependency: whether higher doses might cause a greater effect or whether similar effects might be caused by even lower doses. Such issues should be considered in future studies on vitamin C and childhood asthma.

## Conclusions

We found strong evidence that the effect of vitamin C on asthmatic Egyptian children is heterogeneous. The highest effects observed, the 37% increase in the FEV_1 _level and the 4.2 point increase in the C-ACT level, are substantial and clinically important. It would seem important to carry out further research to confirm our findings and more accurately identify the groups of children who would receive the greatest benefit from vitamin C supplementation.

## Competing interests

This study was not funded by external sources. We have no conflicts of interest.

## Authors' contributions

HH and MB wrote the protocol for the subgroup analysis. MB and AB carried out of the trial which is analyzed in this subgroup analysis. HH wrote the first version of the manuscript and MB and AB participated in the critical revision of the manuscript. All authors read and approved the final manuscript.

## Supplementary Material

Additional file 1 **Additional file contains the protocol that was written before the subgroup analysis was initiated**. Click here for file
